# Association between *MFN2* gene polymorphisms and the risk and prognosis of acute liver failure: a case-control study in a Chinese population

**DOI:** 10.1590/1414-431X20175758

**Published:** 2017-05-15

**Authors:** Y.-L. Wei, Q. Tian, X.-X. Zhao, G.-Z. Qiu, Y. Xu

**Affiliations:** Department of Infectious Diseases, Linyi People's Hospital, Linyi, China

**Keywords:** Acute liver failure, MFN2, Gene polymorphism, Risk, Prognosis, Chinese population

## Abstract

This study aimed to determine the role of *mitofusin 2* (*MFN2*) gene polymorphisms in the risk and prognosis of acute liver failure (ALF). A total of 298 blood samples were collected from 138 ALF patients (case group) and 160 healthy participants (control group). Coagulation function, glutamic pyruvic transaminase (GPT), glutamic oxaloacetic transaminase (GOT), total bilirubin (TB), blood ammonia and lactic acid (LA) were measured. The predictive evaluation of *MFN2* gene polymorphisms in the risk and prognosis of ALF patients was estimated using Kaplan-Meier survival analysis, haplotype analysis, binary logistic regression analysis and Cox regression analysis. Higher levels of GPT, GOT, TB, blood ammonia and LA were observed in ALF patients with the GG genotype of rs873457 or the TT genotype of rs4846085 than in those with the CC genotype of these two SNPs. The GTACAGC and GTGTGGC haplotypes were a protective factor and a risk factor for ALF, respectively. Blood ammonia and LA levels were independent risk factors and the CC genotype of rs873457 and the CC genotype of rs4846085 were protective factors for ALF. ALF patients with the GG genotype of rs873457 or the TT genotype of rs4846085 had a lower survival rate than those with other genotypes of these two SNPs. The rs4846085 and rs873457 polymorphisms were both independent factors affecting the prognosis of ALF patients. *MFN2* gene polymorphisms (rs873457, rs2336384, rs1474868, rs4846085 and rs2236055) may be associated with ALF and the rs873457 and rs4846085 polymorphisms are correlated with the risk and prognosis of ALF.

## Introduction

Acute liver failure (ALF) is defined as severe hepatocyte necrosis and liver injury followed by hepatic encephalopathy within 8 weeks without any pre-existing liver disease (1). ALF often occurs in healthy adults aged approximately 30, and its incidence is approximately 10/1,000,000 per year in developed countries (2). Patients with ALF usually show elevated bilirubin level and transaminase activity and reduced levels of blood coagulation factors, including factor V Leiden and prothrombin. Regarding ALF pathogenesis, viral infection, drug metabolism, cancer, adipose infiltration and irradiation injuries can contribute to abnormal liver cell metabolism, which ultimately results in liver failure (3). A recent report has demonstrated that endogenous factors, including *mitofusin 1* (*MFN1*) and *mitofusin 2* (*MFN2*), are correlated with the occurrence of ALF (4).

The *MFN2* gene encodes a mitochondrial membrane protein that takes part in mitochondrial fusion (5). The MFN2 protein is located on the outer membrane of the mitochondria and has GTPase activity. The mitochondria are the main organelles in charge of energy metabolism and reactive oxygen species generation, and mitochondrial damage may contribute to liver diseases (6). As the *MFN2* gene primarily acts on the regulation of mitochondrial fusion, division, distribution, shape maintenance, and metabolic activity, aberrant *MFN2* gene expression can lead to an increase in oxidative stress, which causes liver cell damage (7). The *MFN2* gene has been shown to be correlated with several liver diseases, including fatty liver and liver failure (8). Previous studies have shown that single-nucleotide polymorphisms (SNPs) in the *MFN2* gene may regulate the function or expression of *MFN2* and that over-expression of MFN2 reduces liver ischemia-reperfusion injury (9,10). Although studies have focused on the relationship between *MFN2* gene polymorphisms and many diseases, such as essential hypertension (11) and axonal Charcot-Marie-Tooth disease (CMT2) (12), its correlation with ALF remains unknown. Therefore, the relationship between *MFN2* gene polymorphisms and ALF has been extensively explored in this study.

## Material and Methods

### Subjects

Blood samples (n=298) were collected from 138 patients with ALF (case group) admitted to Linyi People's Hospital from January 2010 to January 2015 and from 160 healthy participants (control group). Among the patients, there were 112 males and 26 females ranging in age from 20 to 50, and mean age of 37.33±4.94 years. In addition, in terms of pathogenesis, there were 105 suffering from viral hepatitis [8 (7.6%) were infected with hepatitis A virus, 84 (80.0%) with hepatitis B virus (HBV), 7 (6.7%) with hepatitis C virus, 5 (4.8%) with hepatitis E virus (HEV) and 1 (1%) with HBV and HEV]; 22 (21%) suffered from drug intoxication; and 11 (10.5%) had pregnancy-related ALF. All 138 ALF patients received diverse conservative treatments based on the different causes; these treatments included drug therapy such as the use of nucleoside analogues (e.g., lamivudine, telbivudine and entecavir), hormone therapy such as the use of glucocorticoids, nutritional support, therapies that promote hepatocyte regeneration, and oral probiotics or lactulose oral solution to protect the intestinal tract. In addition, 58 patients were treated with plasma-exchange therapy in an artificial liver support system. Diagnostic criteria (13,14) were as follows: acute onset hepatic encephalopathy of grade II to IV (I–IV classification) occurring within 2 weeks and accompanied by the following symptoms: 1) extreme fatigue and severe digestive tract symptoms, including anorexia, lethargy, abdominal distension, nausea and emesis; 2) gradual onset of jaundice; 3) coagulopathy [increased bleeding tendency and prothrombin time <40 s (international normalized ratio (INR) ≥1.5), but other causes that led to uncontrolled gingival bleeding, gastrointestinal bleeding or bleeding hemorrhoids were excluded]; 4) overt conjugated hyperbilirubinemia, elevated aminotransferases (>10,000 IU/U); 5) progressive liver shrinking, and 6) right upper quadrant tenderness. Exclusion criteria included 1) coinfection with other hepatotropic viruses or non-hepatotropic viruses; 2) alcoholic, autoimmune or drug-induced hepatitis; 3) ascites detected by B ultrasound; 4) liver cirrhosis detected by imaging examinations; 5) infection with bacteria or fungi, and 6) history of high blood pressure, heart disease, diabetes, kidney disease or other chronic diseases. A total of 160 healthy individuals were selected as a control group, including 129 males and 31 females ranging in age from 19–55 years, and mean age of 36.82±5.43 years. The basic clinical information of all subjects was obtained, and their coagulation function (using INR), glutamic pyruvic transaminase (GPT), glutamic oxaloacetic transaminase (GOT), total bilirubin (TB), blood ammonia and lactic acid (LA) levels were determined. The study was approved by the Ethics Committee of Linyi People's Hospital and all participants signed an informed consent form.

### DNA extraction and SNP selection

*MFN2* SNPs in the SNP NCBI Database (http://www.ncbi.nlm.nih.gov/sites/entrez?db=Snp) with a frequency over 5% were selected, and tagging SNPs were searched in the HapMap website (http://www.hapmap.org/index.html.en) to determine the SNPs used in the present study. DNA was extracted from blood samples (5 mL) using a Purgene kit (Gentra Systems, USA) according to the manufacturer's protocol and was stored at –20°C. The *MFN2* gene SNPs were analyzed with a SNP genotyping kit purchased from Applied Biosystems (Applied Biosystems Inc., USA). A pair of primers and a TaqMan probe were included in the kit. Seven SNPs were chosen according to previous references: rs2236055, rs4240897, rs1474868, rs2336384, rs873458, rs873457 and rs484608, corresponding to C_15953632_10 (rs2236055), C_26207636_10 (rs4240897), C_1267235_20 (rs1474868), C_11461995_10 (rs2336384), C_8861262_10 (rs873458), C_11461996_20 (rs873457), C_1267226_10 (rs4846085). A 7300 Real-Time PCR System was used for PCR amplification, and the program was set as follows: 95°C for 10 min, followed by 40 cycles of 95°C for 15 s, and 60°C for 60 s (9,11).

### Follow-up

A 24-week follow-up was conducted on all patients after hospital discharge, and the end of follow-up was June 2016. Telephone calls, outpatient services and medical records were utilized to conduct the follow-up, and no patient was lost. Survival time was calculated in weeks, and all the patients, including those who died during hospitalization, were taken into consideration.

### Statistical analysis

All statistical analyses were performed using SPSS 20.0 (SPSS Inc., USA). Data are reported as means±SD, and comparisons between two groups were performed using Student's *t*-test. The Hardy-Weinberg equilibrium test was used for SNP analysis. Binary logistic regression analysis was used to estimate the associations between SNPs and ALF. Haplotype correlation analysis was performed using SHEsis software (http://analysis.bio-x.cn/myAnalysis.php). The survival analysis was conducted using the Kaplan-Meier survival curve method and confirmed by log-rank tests. Patient prognosis was analyzed by Cox proportional hazards survival regression. P*<*0.05 was considered statistically significant.

## Results

### Comparison of baseline characteristics between ALF patients and healthy participants

As demonstrated in Table 1, no significant difference in gender, age or BMI was found between ALF patients and healthy participants. The coagulation function, GPT, GOT, TB, blood ammonia and LA levels in ALF patients were significantly higher than those in the healthy participants (all P*<*0.05).

**Table 1.** Comparison of baseline characteristics between acute liver failure patients and healthy participants.

Characteristic	Normal reference	Control group (n=160)	Case group (n=138)	χ^2^/t	P
Gender (male/female)		129/31	112/26	0.117	0.907
Age (years)		36.82±5.32	37.33±4.94	0.853	0.394
BMI (kg/m^2^)	18.5–24.99	24.37±3.74	25.06±3.59	1.618	0.107
GPT (U/L)	0–40	33.87±5.22	119.86±19.83	52.78	<0.001
GOT (U/L)	8–40	28.69±2.48	151.07±18.81	81.50	<0.001
TB (µmol/L)	3.4–17.1	12.59±2.34	330.34±35.55	112.80	<0.001
Blood ammonia (µmol/L)	20–60	55.06±8.07	87.40±9.81	31.22	<0.001
LA (mmol/L)	0.5–1.7	1.15±0.46	4.96±2.39	19.75	<0.001

Data are reported as mean±SD. BMI: body mass index; GPT: glutamic pyruvic transaminase; GOT: glutamic oxaloacetic transaminase; TB: total bilirubin; LA: lactic acid. The chi-square test or the *t*-test was used for statistical analysis.

### SNP selection of the *MFN2* gene

*MFN2* SNPs were obtained from the NCBI database. The genotype frequencies and theoretical frequencies of the seven SNPs were in accordance with Hardy-Weinberg equilibrium (both P*>*0.05). The *MFN2* SNP selection showed that at rs873457, rs2336384, rs1474868, rs4846085 and rs2236055, the genotype and allele distributions were significantly different between case and the control groups (all P*<*0.05; Table 2), while the rs873458 and rs4240897 SNPs showed no significant difference (both P*>*0.05). At rs873457, the CC genotype and the C allele were more frequent in the control group than in the case group, and the C allele was associated with reduced ALF risk compared with the G allele (P*<*0.05, OR=0.601, 95%CI=0.434–0.833). At rs2336384, the frequencies of the TT genotype and T allele were significantly higher in the control group compared with the case group, and T allele was also associated with decreased ALF risk compared with the G allele (P*<*0.05, OR=0.683, 95%CI=0.494–0.943). For rs1474868, the GG genotype and G allele occurred more frequently in the control group than in the case group, and the G allele was associated with lower ALF risk compared with the A allele (P*<*0.05, OR=0.659, 95%CI=0.478–0.912). At rs4846085, the CC genotype and C allele were more frequently found in the control group than in the case group, indicating that the C allele may be a protective factor for ALF compared with the T allele (P*<*0.05, OR=0.660, 95%CI=0.478–0.913). At rs2236055, the GG genotype and G allele occurred more frequently in the control group than in the case group, and the G allele may lower the risk of ALF compared with the A allele (P*<*0.05, OR=0.663, 95%CI=0.480–0.916).

**Table 2.** Distribution of genotype and allele frequencies of *MFN2* gene polymorphisms in acute liver failure patients and healthy participants.

SNP	SNP/Genotype/Allele	Control group (n=160)	Case group (n=138)	P	OR	95%CI
rs873457						
Genotype	GG	32 (20.0%)	35 (25.4%)		1 (Ref.)	
	GC	65 (40.6%)	76 (55.1%)	0.822	1.069	0.596-1.195
	CC	63 (39.4%)	27 (19.5%)	0.005	0.392	0.203-0.757
Allele	G	129 (40.3%)	146 (52.9%)		1 (Ref.)	
	C	191 (59.7%)	130 (47.1%)	0.002	0.601	0.434-0.833
rs2336384						
Genotype	GG	34 (21.3%)	36 (26.1%)		1 (Ref.)	
	GT	72 (45.0%)	75 (54.3%)	0.955	0.984	0.557-1.739
	TT	54 (33.7%)	27 (19.6%)	0.019	0.458	0.237-0.888
Allele	G	140 (43.7%)	147 (53.3%)		1 (Ref.)	
	T	180 (56.3%)	129 (46.7%)	0.021	0.683	0.494-0.943
rs1474868						
Genotype	AA	29 (18.1%)	35 (25.4%)		1 (Ref.)	
	AG	77 (48.1%)	75 (54.3%)	0.473	0.807	0.449-1.450
	GG	54 (33.8%)	28 (20.3%)	0.013	0.43	0.220-0.841
Allele	A	135 (42.2%)	145 (52.5%)		1 (Ref.)	
	G	185 (57.8%)	131 (48.9%)	0.012	0.659	0.478-0.912
rs4846085						
Genotype	TT	31 (19.4%)	38 (27.5%)		1 (Ref.)	
	TC	80 (50.0%)	75 (54.3%)	0.356	0.765	0.433-1.352
	CC	49 (30.6%)	25 (18.2%)	0.01	0.416	0.212-0.819
Allele	T	142 (44.4%)	151 (54.7%)		1 (Ref.)	
	C	178 (55.6%)	125 (45.3%)	0.012	0.66	0.478-0.913
rs4240897						
Genotype	AA	29 (18.1%)	30 (21.7%)		1 (Ref.)	
	AG	85 (53.1%)	81 (58.7%)	0.786	0.921	0.508-1.669
	GG	46 (28.8%)	27 (19.6%)	0.11	0.567	0.283-1.140
Allele	A	143 (44.7%)	141 (51.1%)		1 (Ref.)	
	G	177 (55.3%)	135 (48.9%)	0.119	0.774	0.560-1.068
rs2236055						
Genotype	AA	27 (16.9%)	35 (25.4%)		1 (Ref.)	
	AG	78 (48.8%)	74 (53.6%)	0.303	0.732	0.404-1.326
	GG	55 (34.4%)	29 (21.0%)	0.008	0.407	0.207-0.798
Allele	A	136 (42.5%)	144 (52.2%)		1 (Ref.)	
	G	188 (58.8%)	132 (47.8%)	0.013	0.663	0.480-0.916
rs873458						
Genotype	TT	20 (12.5%)	24 (17.4%)		1 (Ref.)	
	TC	79 (49.4%)	67 (48.6%)	0.314	0.707	0.359-1.391
	CC	61 (38.1%)	47 (34.0%)	0.217	0.642	0.317-1.300
Allele	T	119 (37.2%)	115 (41.5%)		1 (Ref.)	
	C	201 (62.8%)	161 (58.5%)	0.264	0.829	0.596-1.153

SNP: single nucleotide polymorphism; OR: Odds ratio; CI: confidence interval. Statistical analysis was carried out with the chi-square test.

### Comparison of liver function in ALF patients with different genotypes of *MFN2* polymorphisms

We further analyzed the correlations between different genotypes of these 5 SNPs and liver function indexes. As shown in Table 3, patients with the GG genotype of rs873457 or the TT genotype of rs4846085 had higher coagulation function, GPT, GOT, TB, blood ammonia and LA levels compared with the other genotypes (all P<0.05). There were no significant correlations between liver function indexes and the different genotypes of the other 3 SNPs (all P*>*0.05). All patients had an INR ≥1.5.

**Table 3.** Comparison of liver functions in acute liver failure patients with different genotypes of *MFN2* gene polymorphisms.

SNP/Genotype	GPT (U/L)	GOT (U/L)	TB (µmol/L)	Blood ammonia (µmol/L)	LA (mmol/L)
rs873457					
GG	124.45±18.31	156.75±20.24	348.94±37.27	89.52±7.73	5.5±2.69
GC	124.69±17.21	154.82±16.76	334.66±26.59	90.56±8.25	5.28±2.27
CC	100.33±16.94*	133.12±9.95*	294.09±30.33*	75.74±7.52*	3.38±1.53*
rs2336384					
GG	123.32±14.34	147.61±16.89	330.58±30.81	87.38±10.69	4.41±2.41
GT	117.2±21.37	152.08±19.91	327.53±34.39	86.87±9.92	5.01±2.28
TT	122.65±21.20	152.87±18.12	337.83±44.00	88.89±8.38	5.57±2.56
rs1474868					
AA	116.74±15.15	150.07±21.13	330.13±33.92	88.11±10.42	4.71±2.48
AG	122.11±20.16	151.60±17.12	329.81±38.47	88.07±9.10	5.13±2.43
GG	117.75±23.68	150.88±20.54	332.04±30.10	84.71±10.75	4.83±2.19
rs4846085					
TT	123.76±15.41	152.90±17.84	335.51±28.68	91.86±8.38	4.93±2.31
TC	124.95±18.32	156.05±18.14	339.65±32.84	88.96±8.14	5.50±2.45
CC	98.67±16.44*	133.33±10.15*	294.57±31.24*	75.93±7.79*	3.42±1.54*
rs2236055					
AA	120.04±19.66	153.45±17.20	331.19±28.64	88.32±8.82	4.97±2.35
AG	120.11±20.26	150.58±19.18	330.88±34.66	87.05±10.19	4.91±2.50
GG	118.99±19.57	149.42±20.05	327.95±45.27	87.16±10.21	5.09±2.19

SNP: single nucleotide polymorphism; GPT: glutamic pyruvic transaminase; GOT: glutamic oxaloacetic transaminase; TB: total bilirubin; LA: lactic acid; the first genotype was considered as reference to conduct statistical analysis. Statistical analysis was carried out with one-way ANOVA (*P*<*0.05).

### Correlation analysis between haplotypes of *MFN2* gene polymorphisms and ALF risk

The correlation between haplotypes of *MFN2* SNPs and ALF was analyzed by SHEsis software (Table 4). Haplotypes with frequencies <3% in both groups were not considered. The results showed that among the seven common haplotypes, GTACAGC at rs2236055 was a protective factor for ALF (OR=0.080, 95%CI=0.014–0.443, P*<*0.05), while GTGTGGC at rs873458 was a risk factor for ALF (OR=5.644, 95%CI=1.846–17.258, P*<*0.05). No other haplotypes showed correlations with ALF (P*>*0.05).

**Table 4.** Correlation analysis between haplotypes of *MFN2* gene polymorphisms and the risk of acute liver failure.

Haplotype	Control group (freq)	Case group (freq)	P	OR	95%CI
CGACGGT	2 (0.013)	5 (0.036)	0.148	2.393	0.710–8.068
CGGCGGC	5 (0.031)	3 (0.022)	0.196	0..515	0.186–1.429
CTACAAC	4 (0.025)	5 (0.036)	0.436	1.492	0.543–4.101
CTACGGT	6 (0.038)	3 (0.022)	0.069	0.402	0.147–1.104
CTGCAGC	5 (0.031)	2 (0.013)	0.068	0.348	0.107–1.130
GTACAGC	7 (0.044)	1 (0.007)	<0.001	0.08	0.014–0.443
GTGTGGC	2 (0.013)	10 (0.072)	<0.001	5.644	1.846–17.258

freq: frequency; OR: odds ratio; CI: confidence interval. The haplotypes from top to bottom correspond to rs873457, rs2336384, rs1474868, rs4846085, rs4240897, rs2236055, and rs873458, respectively.

### Binary logistic regression analysis of ALF risk factors

The correlations between *MFN2* gene polymorphisms and liver function indexes with ALF were analyzed by binary logistic regression (Table 5). The results indicated that blood ammonia (P<0.05, OR=1.636, 95%CI=1.364–1.962) and LA levels (P<0.05, OR=10.591, 95%CI=5.364–20.912) were independent risk factors for ALF, while the CC genotype of rs873457 (P<0.05, OR=0.375, 95%CI=0.221–0.634) and the CC genotype of rs4846085 were protective factors for ALF. Other functional parameters, including GPT, GOT and TB (µmol/L), were not associated with ALF (P*>*0.05).

**Table 5.** Binary logistic regression analysis of risk factors for acute liver failure.

Factor	B	SE	Wald	Sig.	OR	95%CI for OR	
						Lower	Upper
Blood ammonia	0.492	0.093	28.099	<0.001	1.636	1.364	1.962
LA	2.36	0.347	46.233	<0.001	10.591	5.364	20.912
rs873457	-0.982	0.269	13.354	<0.001	0.375	0.221	0.634
rs4846085	-0.643	0.277	5.378	0.020	0.526	0.305	0.905

LA: lactic acid; B: partial regression coefficient; SE: standard error; Sig: significance; OR: odds ratio; CI: confidence interval.

### Relationship between *MFN2* gene polymorphisms and short-term prognosis of ALF patients

One hundred and thirty-eight patients were followed-up for 24 weeks (100% follow-up rate). During this period, 83 died, and 55 survived, giving a death rate of 60.15%. The relationship between SNPs of the *MFN2* gene and the risk of ALF was analyzed. The results showed a significantly lower survival rate in ALF patients with the GG genotype of rs873457 than those with the GC + CC genotypes (Figure 1A; P*<*0.05). Patients with the TT genotype of rs4846085 had a remarkably lower survival rate than those with the TC+CC genotypes (Figure 1B; P<0.05).

**Figure 1.** Kaplan-Meier curves of short-term prognosis of acute liver failure patients with different genotypes of *mitofusin 2* (*MFN2*) polymorphisms. *A*, Comparison of survival rates in patients with the GG genotype and GC+CC genotypes of rs873457; *B*, comparison of survival rates in patients with the TT genotype and the TC+CC genotypes of rs4846085.

### Cox proportional hazards survival regression of short-term prognosis of ALF patients

As shown in Table 6, patients' clinical factors and *MFN2* polymorphisms were introduced into a Cox regression model. The results showed that GPT, GOT, TB, blood ammonia and LA were not associated with the prognosis of ALF patients (all P*>*0.05), but the rs4846085 and rs873457 polymorphisms were both independent factors affecting the prognosis of ALF patients (all P*<*0.05).

**Table 6.** Cox proportional hazards survival regression of short-term prognosis of acute liver failure.

Factor	B	SE	Wald	Sig.	OR	95%CI for OR	
						Lower	Upper
GPT (U/L)	0.005	0.005	0.701	0.402	1.005	0.994	1.015
GOT (U/L)	-0.001	0.006	0.045	0.831	0.999	0.987	1.01
TB (µmol/L)	-0.004	0.004	1.509	0.219	0.996	0.989	1.003
Blood ammonia (µmol/L)	0.012	0.012	0.933	0.334	1.012	0.988	1.036
LA (µmol/L)	0.017	0.046	0.145	0.703	1.018	0.93	1.113
rs873457	-0.669	0.234	8.174	0.004	0.512	0.324	0.81
rs4846085	-0.663	0.233	8.084	0.004	0.515	0.326	0.814

GPT: glutamic pyruvic transaminase; GOT: glutamic oxaloacetic transaminase; TB: total bilirubin; LA: lactic acid; B: partial regression coefficient; SE: standard error; Sig: significance; OR: odds ratio; CI: confidence interval.

## Discussion

The findings of this study revealed that *MFN2* gene polymorphisms (rs873457, rs2336384, rs1474868, rs4846085 and rs2236055) might be associated with ALF and that the rs873457 and rs4846085 polymorphisms are correlated with the risk and prognosis of ALF.

In this study, we selected seven SNPs of the *MFN2* gene in ALF patients and analyzed the relationship between *MFN2* SNP allele distribution, haplotype and ALF. The results indicated that rs873457, rs2336384, rs1474868, rs4846085 and rs2236055 were closely correlated with ALF. Current opinions suggest that if a disease-related mutation is located in the non-coding region, the mutation would function by regulating the transcription of the gene instead of affecting the translation of the gene (15). In our study, rs873457, rs2336384, rs1474868, rs4846085 and rs2236055 were all located in the transcriptional regulatory region of *MFN2*. To be more specific, they were located at the TATA box, the CCAAT box and the start of transcription at the second intron, which is in charge of regulating the transcription of *MFN2*. *MFN2* gene transcription might be down-regulated when mutations occur at these SNPs, which might lead to the malfunction of mitochondria (16). Mitochondria are often called “the powerhouse of the cell” because they generate most of the cell's supply of adenosine triphosphate (ATP). The amount of ATP determines the responsiveness of the cell toward stimuli, and cells will undergo severe damage due to the lack of ATP. Currently, it is believed that the decreased level of *MFN2* gene expression leads to the malfunction of mitochondria and increases in the ROS levels in the cell, which result in liver cell damage and ALF (17). Decreased expression of the *MFN2* gene also leads to RAS-mediated PI3K/Akt activation, which results in abnormal cell cycle progression and malfunctions in multiple organs (18). Moreover, the concentration of Ca^2+^ is believed to play a critical role in oxidative metabolism, and when down-regulating the expression of the *MFN2* gene, Ca^2+^ in the mitochondria accumulates, which leads to the elevation of oxidative stress and cell damage (19).

By comparing liver functions and different genotypes at rs873457 and rs4846085, the CC genotype was found to contribute to the decrease of liver function indexes, while patients with the GG genotype of rs873457 or the TT genotype of rs4846085 had higher coagulation function, GPT, GOT, TB, blood ammonia and LA levels. However, at rs2336384, rs1474868 and rs2236055, the variation of genotypes did not affect liver function significantly. We presume that the mechanism by which rs873457 or rs4846085 affects liver function may have to do with their location in the *MFN2* gene intron, which is responsible for the transcriptional regulation of the *MFN2* gene (11). The liver is the main organ in charge of metabolism in the human body; therefore, liver injury results in the elevation of coagulation function, GPT and GOT (20). Moreover, the liver is also responsible for urea and lactate metabolism, and a large area of damage in the liver also results in the elevation of blood ammonia and lactate levels (21). Therefore, multiple indexes could be used in the evaluation of liver function and ALF patient prognosis. These results were consistent with our analyses, which demonstrated that the rs873457 or rs4846085 CC genotypes are protective factors for ALF. Patients with the rs873457 GG genotype or the rs4846085 TT genotype have lower survival rates, indicating that the rs873457 or rs4846085 polymorphisms may be independent factors that correlate with ALF risk and prognosis.

The haplotype analysis demonstrated that GTACAGC was a protective factor for ALF, while GTGTGGC was a risk factor for ALF. Other haplotypes of the *MFN2* gene and their relationships with ALF still remain unclear. Haplotype analysis has been valued as a good method in genetic studies of complex diseases with multiple variants, and this consensus may lead to the development of a more efficient strategy to identify genetic variants that increase the risk of human diseases (22). Moreover, Wang et al. (11) verified that *MFN2* haplotypes were risk factors for hypertension, which suggests that SNP haplotypes of the *MFN2* gene may also be correlated with other diseases.

ALF is a fatal disease that is associated with the rapid arrest of normal hepatic function, and is one of the most challenging emergencies encountered in clinical practice. Presently, effective prevention and therapy against ALF are not available but are urgently needed. The positive relationship between *MFN2* gene polymorphisms and the occurrence of ALF will provide a new genetic tool to identify groups at high risk for ALF and shed light on the early prediction of ALF patients and the prevention of this disease.
